The article "Multiscale Convolutional Neural Networks with Attention for Plant Species Recognition" was published in 2021. Journal: Comput Intell Neurosci.

# Multiscale Convolutional Neural Networks with Attention for Plant Species Recognition

**DOI:** 10.1155/2021/5529905

**Published:** 2021-07-05

**Authors:** Xianfeng Wang, Chuanlei Zhang, Shanwen Zhang

**Affiliations:** ^1^School of Information Engineering, Xijing University, Xi'an 710123, China; ^2^College of Artificial Intelligence, Tianjin University of Science and Technology, Tianjin, 300222, China

## Abstract

Plant species recognition is a critical step in protecting plant diversity. Leaf-based plant species recognition research is important and challenging due to the large within-class difference and between-class similarity of leaves and the rich inconsistent leaves with different sizes, colors, shapes, textures, and venations. Most existing plant leaf recognition methods typically normalize all leaf images to the same size and then recognize them at one scale, which results in unsatisfactory performances. A novel multiscale convolutional neural network with attention (AMSCNN) model is constructed for plant species recognition. In AMSCNN, multiscale convolution is used to learn the low-frequency and high-frequency features of the input images, and an attention mechanism is utilized to capture rich contextual relationships for better feature extraction and improving network training. Extensive experiments on the plant leaf dataset demonstrate the remarkable performance of AMSCNN compared with the hand-crafted feature-based methods and deep-neural network-based methods. The maximum accuracy attained along with AMSCNN is 95.28%.

## 1. Introduction

Plants are the life forms with the largest number of species and the most extensive distribution on Earth and directly affect the ecological system on which human beings live. Plants are also important resources for human survival and development, essential resources for human production and life, and the basis for human survival. With the disappearance of a lot of plant species, people have realized the importance of protecting plant species diversity. To protect plants, the first step is to identify plant species, which can be achieved by their leaf, fruit, seed, branch, flower, skin, and so on. How to quickly recognize an unknown plant without the related professional knowledge is a huge challenge, because plant leaves are highly diverse and inconsistent. With the development of image processing, pattern recognition, computerization, Internet, and big data, many various approaches have been presented to implement plant species classification systems. Plant species have rich leaves in most of a year, and a leaf has abundant classification features such as leaf margin, vein, skeleton, and fissure depth, which are the main basis whether for plant morphology or automatic methods to recognize plant species. Automatic plant classification can be achieved by extracting features from its leaves. However, due to the variation, irregularity and large within-class difference of the plant leaf shape and texture comparing to the industrial parts, as shown in Figure 1, the leaf-based plant species recognition is one of the challenging researches. From Figure 1, it is seen that the different plants leaves vary greatly and have different sizes, textures, shapes, venation, and disorder. Moreover, it is known that in different growth conditions or different shooting distances, even for the same species, plant leaves still have different sizes [1, 2], as shown in Figures 1(c) and 1(d).

The feature extraction of plant leaf image is a crucial step of a plant recognition method. There are many plant species recognition algorithms [1–5], which can be divided into two main types of feature representation methods for describing leaf images, i.e., hand-crafted features [6, 7] and deep learning features [8, 9]. In fact, the hand-crafted features are mainly dependent on the ability of computer vision experts to encode the morphological characters of the leaves [2–6]. The classical predefined feature extraction-based approaches rely mainly on the features and classifier or select certain leaves within a dataset to achieve high accuracy rates. But it is very difficult to select the optimal hand-crafted features due to the various leaves and the different species with similar shape and texture characteristic [10, 11]. Furthermore, most of the existing plant species recognition systems rely on a lot image preprocessing steps and human intervention to select certain points of the leaf to help the system align and normalize the leaf images or to select the best result among a few candidates after the classification is done. The hand-crafted feature extraction is a complex, time-consuming process which needs to be altered whenever the problem or the dataset changes.

The deep-learning-based methods are able to automatically learn the classification features from the input leaf images without the complex image preprocessing. AlexNet, ResNet, and VGG16 are three classical CNN models [12]. AlexNet contains 650,000 neurons, five convolution layer, three pooling layers, and three fully connected layers. ResNet has a residual unit to transmit the original input data directly to the back of the layer. VGG16 improves the relationship between the depth of CNN and its performance, repeatedly stacking the small convolutional kernel of 3 × 3 and the maximum pooling of 2 × 2 to construct the CNN with the depth of 16–19 layers.

Recently, deep-learning-based plant recognition methods have gotten more and more attention, and several deep learning models have been constructed for plant identification and achieved perfect accuracy [13]. To improve the plant recognition ability in the complex environment, Zhu et al. [14] proposed an improved deep convolutional neural network (CNN) by taking advantage of the Inception V2 with batch normalization instead of the convolutional neural layers in faster region-based CNN (RCNN). The experimental results show that the proposed approach has higher recognition accuracy than faster RCNN in recognizing leaf species in the complex background. Zhu et al. [15] proposed a deep CNN-(DCNN-) based plant identification method. DCNN consists of 16 convolutional layers followed by 5 max pooling layers, 3 fully connected layers, and a final SoftMax layer. The experiments on several plant datasets validated the remarkable performance of the very deep neural network compared to the hand-crafted features.

From the above CNN-based plant recognition methods, it is concluded that the performance of the CNN models rely on several factors including availability of large dataset, more computing power and new ideas and algorithms. Convolutional layers automatically learn the kernel parameters from the training images to extract local features from the original images. It is very crucial to choose the size of convolutional kernels for feature extraction in CNN. The kernels with small size can extract short edges or low-frequency feature, while the high-frequency feature or the other suitable feature of the images cannot be extracted at the same time. Similarly, the kernels with large scale can extract more big features but without having low-frequency feature of the images. If every convolutional layer uses the same filter size or even alternative size, CNN deeper and complex computations make training slow. Considering multiscale features, Du et al. [16] and Rasti et al. [17] proposed two multiscale CNN (MSCNN) models, which consist of multiple different scale feature learning modules. The main difference between the two models is that the multiscale features learned by the first model are fused at one interfusion layer, while by the second model are step-by-step fused. Hu et al. [18] proposed a multiscale fusion CNN (MSFCNN) for plant leaf recognition at multiple scales. Along with the depth of MSFCNN, multiscale images are progressively handled and the corresponding features are fused.

The attention mechanism is widely used in a lot of computer vision, image processing, and deep learning [19, 20], which can make full use of the local and global features of the samples, assign higher weight to important features, highlight the impact of key input information on the model output, and then teach systems to pay attention to important information and ignore irrelevant information. Li et al. [21] developed a multibranch CNN with attention (MBCNNA) for plant species recognition. MBCNNA consists of 12 convolutional layers, 4 max pooling layers, and 2 fully connected layers. The first part of MBCNNA is an attention block to reduce the influence of background, while the latter part is multibranch CNN to extract the multiview features through multichannel. Zhu et al. [22] proposed a plant species recognition method based on DCNN with two-way attention model. The first attention way aims to recognize the plant species, while the second attention way focuses on the discriminative features of the input image by finding the max-sum part of the fully convolutional network heat map.

Inspired by MSCNN [16–18] and attention mechanism [19–22], a modified MSCNN with attention (AMSCNN) model is constructed for plant species recognition. The contributions of the proposed method are given as follows:

1. Multiscale convolution is used to learn the low-frequency and high-frequency features of the input images
2. Attention mechanism is utilized to capture the rich contextual relationships for better feature extraction and improvement of the network training
3. Extensive experiments are conducted to validate AMSCNN

The remainder of this paper is organized as follows.  Section 2 overviews the classical CNN and multiscale convolution. AMSCNN is introduced in Section 3.  Section 4 presents experiments and experimental results. Finally, Section 5 discusses the proposed method and concludes this paper.

## 2. Related Works

### 2.1. Plant Identification by Texture, Shape, and Color Features (TSC)

Plant species can be identified by texture, shape, and color of its leaf (TSC) [10]. First extract the features of texture, shape, and color of each leaf. Then combine three kinds of features as a feature vector. Finally, the SVM classifier is applied to leaf classification. This method is a classical hand-crafted feature extraction-based method.

### 2.2. CNN and VGG16

CNN stands out from the traditional neural networks (NN) in two characteristics, sparse connection and weight sharing, which can reduce the number of parameters and prevent overfitting. The basic architecture of CNN consists of four kinds of layers, namely convolutional layer, pooling layer, fully connected layer, and classification layer. VGG network can explore the relationship between the depth of CNNs and their performance [23]. Each block is made by several consecutive 3 × 3 convolutions and followed by a max-pooling layer. VGG16 is a classical CNN model [24], containing 13 convolutional layers, 5 pooling layers, 3 fully connected layers, and a classification layer. It is simple but contains a large number of model parameters, which result in a lot of training time to adjust these parameters. Increasing network depth can improve network classification ability, but only deepening the network depth is likely to cause gradient explosion or gradient vanishing. The architectures of CNN and VGG16 are shown in Figure 2.

### 2.3. Residual Neural Network (ResNet)

ResNet is used to solve the problems of gradient disappearing or explosion during training very deep CNN model [23]. It outperforms the classical CNN models at a variety of tasks, such as object detection and semantic image segmentation. Compared with the ordinary network block, the ResNet block mainly adds a path between the input and output, so that the network only needs to learn the residual of multilevel resolution features. The architecture of ResNet block is shown in Figure 3, where *x*_*i*_ and *x*_*i*+1_ are the input and output of the *i*th layer, *F*(.) and *f*(.) are residual and activation functions, respectively.

### 2.4. Multiscale Convolution (MSC)

MSC can extract the multiscale features, containing several MSC blocks. Each block consists of MSC layer and a flat convolutional layer, as shown in Figure 4(b) [17, 18].

## 3. Multiscale CNN with Attention

Inspired by MSCNN [17, 18] and attention mechanism [19, 20], a MSCNN with attention (AMSCNN) based plant species recognition method is proposed. The architecture of AMSCNN is shown in Figure 5. After multiscale convolutions of 3 × 3,5 × 5 and 7 × 7, attention is employed to make the spatial variation robustness of the input data stronger. Different levels of features are fused to improve the model's ability to express image semantic features, and SoftMax classifier is used for plant recognition in the output decision layer. Different from MSCNN, AMSCNN utilizes the attention mechanism to capture rich contextual relationships for better feature representations and decrease the size of training and model parameters. MSC block has three convolutional operations with different kernel sizes, as shown in Figure 5(b). MSC within the same layers of CNN helps the model to secure low-frequency and high-frequency details of the original images.

### 3.1. CNN Part

CNN part uses a single-size convolutional kernel and single-channel mode to extract feature from the input image, while extracting and enhancing feature information in the form of alternating convolution and pooling operations. Max pooling layer is applied to filter the extracted features by selecting the maximum value of each filter and then reduce the dimensionality. The convolution operation is output by the feature map of the current layer after the activation function. The calculation formula for the convolution layer is as follows:

(1) $$\begin{array}{c} x_{j}^{l}=f\left(\sum_{i=M_{j}}x_{i}^{l-1}\times k_{i}^{l}+b_{j}^{l}\right), \end{array}$$

where *k* is the convolution kernel, *M*_*j*_ is the input feature, and *b* is the bias value.

The pooling operation is a form of nonlinear downsampling, which can reduce the size of the feature maps extracted from the convolutional layers to achieve spatial invariance. The operation leads to faster convergence and improves the generalization performance [8, 9]. When the feature map *x*_*j*_^*l*^ is passed to the pooling layer, the pooling operation is applied to the feature map *x*_*j*_^*l*^, which produces a pooled feature map *x*_*j*_^*l*+1^ as the output. The max pooling and average-pooling operations are often used, which are calculated respectively as follows:

(2) $$\begin{array}{c} x_{j}^{l+1}=\underset{i\in R_{j}}{\max}x_{j}^{l},\\ x_{j}^{l+1}=\underset{i\in R_{j}}{\text{average}}x_{j}^{l}, \end{array}$$

where *R*_*j*_ is the *j*^th^ pooling region in feature map *x*_*j*_^*l*^ and *i* is the index of each element within it.

The convolution operation is used to extract feature maps, while the pooling operation is to adjust the size of feature maps without changing the number of the feature maps.

In general, the nonlinearity activation function ReLU (Rectified Linear Units) is used in the middle full-connection layer. The mathematical expression is as follows:

(3) $$\begin{array}{c} f\left(x_{j}^{l}\right)=\max\left(0,x_{j}^{l}\right), \end{array}$$

where *x*_*j*_^*l*^ is the feature map in the *l*th layer.

### 3.2. MSC Part

The output feature map of the *l*th MSC layer with depth can be calculated as [16–18]

(4) $$\begin{array}{c} F_{m}^{l}=\max\left(0,\mathrm{concat}\left(f_{1}^{l},f_{2}^{l},f_{3}^{l}\right)\right), \end{array}$$

where *f*_1_^*l*^, *f*_2_^*l*^, *f*_3_^*l*^ are the feature maps obtained after MSC calculated as *f*_1_^*l*^=*w*_1_^*l*^*F*_*l*−_^1^+*b*_1_^*l*^, *f*_2_^*l*^=*w*_2_^*l*^*F*_*l*−_^1^+*b*_2_^*l*^, *f*_3_^*l*^=*w*_3_^*l*^*F*_*l*−_^1^+*b*_3_^*l*^, *w*_*i*_^*l*^(*i*=1,2,3) is a convolutional filter, and *b*_*i*_^*l*^(*i*=1,2,3) is bias.

Three filters *w*_*i*_^*l*^(*i*=1,2,3) with sizes 3 × 3,5 × 5 and 7 × 7 are utilized to convolve with *F*_*l*−_^1^ feature map. *b*_*m*_^*l*^ is added to each feature map of the *l*^th^ MSC layer. Each convolution operation is output in feature maps and then they are merged by concatenating along the spectral dimension. The next layer of MSC is 3 × 3 convolutional layer to reduce the spectral dimension of feature maps. To facilitate gradient flow in the training process of the network, a skip connection is used after every two layers.

### 3.3. Attention Part

Attention mechanisms teach systems to pay attention to focus on important information and ignore irrelevant information. Suppose that the convolution kernel that inputs the attention structure is *X*, and it is retained as one of the inputs of the residual branch, *X* ∈ *ℝ*^*H*×*W*×*C*^. *H*, *W*, and *C* represent the length, width, and number of channels of the feature map. It is then sent to two separate branches for two different types of pooling operations. Let the global average-pooling process be *F*_avg_ and the global maximum pooling process be *F*_max_ and the outputs of *F*_avg_ and *F*_max_ be Att_avg_ and Att_max_, the Att_avg_ ∈ *ℝ*^1×1×*C*^, and Att_max_ ∈ *ℝ*^1×1×*C*^. The one-dimensional weight sequence Att_max_ can filter out the global background information of the target object, while Att_max_ can highlight the saliency of the target object. Let *X*=[*x*_1_, *x*_2_,…, *x*_*m*_], where *x*_*c*_ represents the parameters of the *c*th convolution kernel. The calculation relation is as follows:

(5) $$\begin{array}{c} \mathrm{At}t_{\mathrm{avg}}=\frac{1}{H\times W}\sum_{i=1}^{H}\sum_{j=1}^{W}x_{c}\left(i,j\right)=F_{\mathrm{avg}}\left(x_{c}\right), \end{array}$$

(6) $$\begin{array}{c} \mathrm{At}t_{\max}=\mathrm{argmax}\left(\sum_{i=1}^{H}\sum_{j=1}^{W}x_{c}\left(i,j\right)\right)=F_{\max}\left(x_{c}\right). \end{array}$$

These two kinds of attention maps are input into 1 × 1 convolution and then are fused in a cascade way to generate attention map of the entire spatial information as follows:

(7) $$\begin{array}{c} \mathrm{Att}=\delta \left(\mathrm{Con}v_{1\times 1}\left[F_{\mathrm{avg}}\left(x_{c}\right);F_{\max}\left(x_{c}\right)\right]\right),\\ F=X⊗\mathrm{Att,} \end{array}$$

where *δ* is Sigmoid activation function, Conv_1×1_ is to fuse two pooling operations with the size of 1 × 1 kernel, [] is a cascading operation, and *F* is the attention weighted feature map.

The attention feature is obtained by adding the channel-wise representation and space-wise representation:

(8) $$\begin{array}{c} \mathrm{outpu}t_{\mathrm{ch}}=\mathrm{outpu}t_{\mathrm{avg}}+\mathrm{outpu}t_{\max}, \end{array}$$

where output_avg_ and output_max_ are the channel-wise representation and space-wise representation, respectively.

### 3.4. Fusion Part

As mentioned earlier, the multiscale feature extraction module allows the network to result in a similar type of feature maps of each input image. In order to fuse the corresponding level of features from each source image, the extracted features are merged together by feature fusion concatenation operation as

(9) $$\begin{array}{c} F_{M}=\mathrm{Concat}\left(f_{1}^{m},f_{2}^{m}\right), \end{array}$$

where *f*_1_^*m*^ and *f*_2_^*m*^ are the feature maps obtained by feature extraction from two original images *I*_1_ and *I*_2_, respectively, and *F*_*m*_ is the fused feature representation. Later, this fused image representation is utilized in the reconstruction module as an input for the restoration of the fused image.

The simple fusion method is to concatenate the results of MSC layer and flatten them in order to feed it to the classification module.

### 3.5. Activation Part

Two fully connected layers use ReLU to model the abstract representation of the leaf feature maps, which is calculated as follows:

(10) $$\begin{array}{c} f_{re}=\mathrm{ReLU}\left(WX+b\right). \end{array}$$

### 3.6. Classification Part

The plant recognition task is implemented by the SoftMax classifier. Its objective function is formulated as follows:

(11) $$\begin{array}{c} J\left(W\right)=-\frac{1}{N}\sum_{n=1}^{N}\sum_{c=1}^{C}\ell \left(y_{n}==c\right)\log\frac{\exp\left(W_{c}^{T}X_{i}\right)}{\sum_{p=1}^{C}\exp\left(W_{p}^{T}X_{i}\right)}, \end{array}$$

where (*X*_*i*_, *y*_*i*_)(*i*=1,2,…, *N*) is the training set, *X*_*i*_ is an *i*th training sample, and *y*_*i*_ is a the corresponding label. *N* and *C* are the numbers of training samples and classes, and *ℓ*(*∗*) is an indicator function.

Equation (11) is incorporated with the proposed AMSCNN architecture and is optimized by using the stochastic gradient descent algorithm, and the deep learning toolbox is MatConvNet.

Gradient descent algorithm is adopted for optimization, and the weight of gradient descent is updated as

(12) $$\begin{array}{c} W_{\mathrm{new}}=W_{\mathrm{old}}-\eta \frac{\partial E}{\partial W_{\mathrm{old}}}, \end{array}$$

where *W*_old_ and *W*_new_ are weights before and after updating, respectively, *η* is the learning rate, and *E* is the composite function of weight *W*.

## 4. Experiments and Analysis

AMSCNN is applied to plant recognition, validated on a public plant leaf image database named ICL, and compared with three classical CNN models (AlexNet, ResNet, and VGG16), three CNN-based plant species identification methods (DCNN [15], MSFCNN [18], and MBCNNA [21]), and a classical hand-crafted feature extraction-based method, i.e., plant leaf type detection using texture, shape, and color features (TSC) [10].

### 4.1. Dataset and Augmentation

ICL database was constructed by the intelligent computing laboratory of Chinese Academy of Sciences in 2005. It has 17032 plant leaf images from 220 species and the image number of each class is unequal.  Figure 6 shows some leaf images from ICL dataset. From Figure 6, it is known that the leaf images of ICL set are various and complex with large within-class difference and large between-class similarity, and the sizes and shapes of leaves are irregular.

For plant species with fewer leaf images, each leaf image is augmented through some simple extension methods. Each image is rotated by 45° at each time to generate 4-fold images, bilinear interpolation is adopted to fix images to the pixel size of 450 × 750, and salt and pepper noise is also added to the images to ensure the validity of leaf images, which randomly changes pixel values in the images, whitening some pixel points and blackening some other pixel points. From augmentation processing, each original leaf image can be augmented to more than 50 images.  Figure 7 shows 27 augmented images of a leaf image of Flower of Hedge Glorybind.

### 4.2. Experiments and Results

The code environment is Win10 + CUDA + VS + Anaconda + Keras configuration GPU, the memory is 96 G, and the development environment is PyChARM. Keras is highly modular, simple, and scalable, allowing seamless switching between CPU and GPU. The experiments are performed on an Ubuntu workstation equipped with an Intel (R) Xeon (R) CPU E5-2650 v4 @2.40 GHz, NVIDIA 1080ti GPUs with 3,584 CUDA cores, and 11 GB of HBM2 memory. The core frequency is up to 1,328 MHz and the floating point performance is 10.6 TFLOPS. The constructed AMSCNN model is implemented in MatConvNet, Python 3.5.2, and TensorFlow-GPU 1.8.0. The size of the input image is 224 × 224, and the value of batch size is set to 50. The bias vector and weight matrix are set randomly. The number of iterations is set to 30,000. The momentum is set to 0.9. The learning rate is originally set 0.95 and becomes half of the original per 300 iterations. The overfitting is reduced by using stochastic gradient descent momentum method with a weight decay value of 0.0001 and a momentum value of 0.9.

In order to indicate the superiority of AMSCNN, an image with no background and an image with background are used as test samples to input AMSCNN. The feature maps of the different convolutional layers are shown in Figure 8. From Figure 8, it is seen that AMSCNN can extract the deep discrimination features, and the attention mechanism enables the network to focus on plants and reduce the impact of background factors. After attention block, the background is filtered while the branches and leaves of the plants are retained, as shown in Figure 8(e).

Several plant species recognition experiments are performed on the original ICL leaf image dataset by 5-fold-cross validation and the AMSCNN with AlexNet is compared, ResNet and VGG16. The numbers of images considered in the following experiments with the resized dimension are shown in Table 1.

The results are shown in Table 2.

From Table 2, it is seen that the recognition rate of AMSCNN is the highest, but all recognition rates of four CNN models are very low. The reason is the serious imbalance of the number of experimental dataset. In ICL dataset, the image number of each species is unequal from 26 to 1078.

We augment the original dataset so that each species has more than 500 leaf images and then obtain an augmented dataset. In the following experiments on the augmented dataset of ICL, 5-fold-cross validation is adopted for testing the effectiveness of the proposed method.  Figure 9 is the accuracy rates of four CNN models versus the number of iterations. From Figure 9, it is found that in the model training process the recognition performance of the four models continues to improve with increasing the iterations, and AMSCNN outperforms the other models, and after 1500 iterations, the recognition rates of DCNN, MSCNN, and MCNNA become slower, while the recognition rate of AMSCNN is still increasing, which indicates that the training performance of AMSCNN is relatively stable without fluctuation.

The plant species recognition rates of five methods are shown in Table 3.

From Figure 8 and Table 3, it is found that four CNN-based plant species recognition methods have better training effect and higher detection accuracy compared to the classical TSC-based method, and AMSCNN outperforms consistently. The possible reason is that CNN can effectively extract the high-level features from the complex leaf image and avoid complex image preprocessing. In CNN, the basic features are extracted by the lower convolutional layer, and the more abstract the features extracted by the higher convolutional kernel are, the more shape characteristic of the leaf image can be reflected. The proposed AMSCNN carries out multiscale convolution on the features extracted from the fourth convolutional layer and then performs feature fusion with attention mechanism, so as to improve the AMSCNN performance to describe the leaf image. In AMSCNN, more variation in the dataset being considered could be helpful to enhance the recognition accuracy. AMSCNN combines low-level features with more abstract high-level features to discover estimable relationships in mass leaf image dataset.

## 5. Conclusions

With the development of computer vision, plant species identification based on deep learning methods can be effectively carried out. In view of the various shapes and sizes of the plant leaves and the large number of the weight parameters of CNN, a multiscale CNN with attention (AMSCNN) model was constructed for enhancing ability of the multiscale feature extraction and was applied to the plant species identification. The experimental results on the public leaf image dataset validated that the proposed method is effective and feasible. By comparing with the existing deep learning models, AMSCNN uses multiscale convolution and iteration to capture pairwise feature interactions for image classification and utilizes the attention mechanism to learn the critical area and fine-grained feature, which can accelerate the convergence of the network. From Tables 2 and 3, it is found that the unbalance of leaf image number seriously affects the performance of CNN model. So it is necessary to respond to the imbalance problem of dataset. Further work can be done on evaluating deep learning for feature learning, as well as the use of dissimilarity feature space, since the number of plant species is huge. We will further develop it to deeper networks and study its performance on the larger leaf image dataset.

## Figures and Tables

**Figure 1:** Plant leaves in different seasons, illuminations, and different attitudes. (a) 10 species leaves with very different shapes, (b) 10 different species leaves with very similar shape, (c) 10 Aesculus leaves with different shapes, and, (d) 10 *Fraxinus chinensis* leaves with different sizes and locations.

**Figure 2:** The architectures of CNN and VGG16. (a) CNN and (b) VGG16.

**Figure 3:** The architectures of ResNet.

**Figure 4:** Difference between the basic convolutional layer of CNN and multiscale convolutions. (a) Convolutional layer with one convolution and (b) convolutional layer with MSCs.

**Figure 5:** The architecture of AMSCNN. (a) The component modules of AMSCNN and (b) MSC.

**Figure 6:** Plant leaf image samples. (a) Some kinds of plant leaf images with large between-class difference. (b) Some kinds of plant leaf images with large between-class similarity. (c) 14 original cherry blossom leaf images with at different scales, colors, and shapes.

**Figure 7:** One original leaf image and its 27 augmented leaf images. (a) Original leaf image, (b) 18 augmented leaf images with different angles and shapes, and (c) 9 augmented leaf images with different scales.

**Figure 8:** Some examples of feature maps and convolutional kernel. (a) Two original leaf images, one without background and one with complex background, (b) feature maps of the first convolutional layer, (c) convolutional kernels of the first convolutional layer, (d) feature maps of the 5th convolutional layer, and (e) feature maps of the attention layer.

**Figure 9:** The accuracy rates of four CNN models versus the number of iterations.

**Table 1:** The number of images.

	Original images	Augmented images	Training images	Test images
Number	17032	861600	691280	170320
Size	450 × 750 × 3	450 × 750 × 3	224 × 224 × 3	224 × 224 × 3

**Table 2:** Recognition rates of four CNN models.

Method	AlexNet	ResNet	VGG16	AMSCNN
Accuracy	68.53	71.12	67.48	73.62

**Table 3:** Recognition rates of 4 plant species recognition methods.

Method	TSC	DCNN	MSCNN	MCNNA	AMSCNN
Accuracy	89.83	93.54	94.16	94.75	95.28

## Data Availability

The dataset used in this study is available at https://pan.baidu.com/s/1UfYnApJuVB-PklWRxJRc7g (extraction code: dtlk).
